The article "Levetiracetam Attenuates the Spinal Cord Injury Induced by Acute Trauma via Suppressing the Expression of Perforin" was retracted in 2022. Reason: concerns about the peer review.

# Levetiracetam Attenuates the Spinal Cord Injury Induced by Acute Trauma via Suppressing the Expression of Perforin

**DOI:** 10.1155/2022/7218666

**Published:** 2022-05-19

**Authors:** Hong Xia, Jiaqiang Huang, Jian Liu, Hua Zhang, Dawei Chen, Wen Zhang, Xianghong Zhou, Zhouyang Wei, Zhaoxiang Liu

**Affiliations:** ^1^Trauma Center of Xiangtan Central Hospital, 411100 Xiangtan City, Hunan Province, China; ^2^Department of Orthopedics, Xiangtan Central Hospital, 411100 Xiangtan City, Hunan Province, China; ^3^Intensive Care Unit of Surgery, Xiangtan Central Hospital, 411100 Xiangtan City, Hunan Province, China; ^4^Biomedical Transformation Research Institute of Zhuhai People's Hospital, 519000, Zhuhai City, China; ^5^Department of Spine Surgery, Xiangtan Central Hospital, 411100 Xiangtan City, Hunan Province, China; ^6^Prehospital Emergency Department of Xiangtan Central Hospital, 411100 Xiangtan City, Hunan Province, China; ^7^Department of General Medicine, Xiangtan Central Hospital, 411100 Xiangtan City, Hunan Province, China

## Abstract

The spinal cord injury (SCI) is one of the major reasons causing the motor dysfunctions of the patients. At present, few therapeutic strategies can effectively improve the symptom of SCI. Levetiracetam has been confirmed to alleviate the injury of nerve cells, while its functions in SCI remains unclear. In this study, C57BL/6J mice were used to establish SCI models to observe the effect of levetiracetam on SCI. The mice were fed with 180 mg/kg levetiracetam when suffering from SCI, and Basso mouse score (BMS) and CatWalk-assisted gait analysis were used to observe the motor functions of the mice. Nissl staining and TUNEL staining were used to observe the injury of nerve cells. The abundance of inflammatory factors was measured by ELISA. The permeability of blood-spinal cord barrier (BSCB) in mice was detected with macrophage infiltration analysis. Moreover, the abundance of perforin in the tissues was detected by western blot. The results showed that the SCI mice treated with levetiracetam exhibited lighter motor dysfunction compared with the mice treated with saline. Levetiracetam can effectively reduce the inflammatory reactions and alleviate apoptosis of the nerve cells. Moreover, levetiracetam remarkably decreased the BSCB permeability of SCI mice. Besides, it was also found that levetiracetam can significantly inhibit the expression of perforin. In conclusion, this study suggests that levetiracetam can attenuate the injury of BSCB to block the progression of SCI via suppressing the expression of perforin.

## 1. Introduction

The spinal cord injury (SCI) has been widely accepted as a key reason for the disability of the patients [1, 2]. The injury in spinal cord nerve has been proved as a biomarker event for the patients suffering from SCI, which may induce the disability of the motor function [3]. Blood-spinal cord barrier (BSCB) plays an important role in preventing the neuronal injury induced by inflammatory reactions, and the disruption of BSCB may aggravate the secondary injury of the spinal cord [4, 5]. The study has indicated that the poor outcomes of SCI patients are associated with the injury of BSCB [6]. Due to the low regenerative ability of nerve cells, healing neural injury-related disease has become an intractable question in clinical treatment [7, 8]. At present, even with the current techniques, the prognosis of the patients with spinal injury remains unsatisfactory [9]. Thus, preventing the injury induced by inflammatory stress has been widely accepted as a promising strategy for improving the spinal cord injury.

The article "Levetiracetam Attenuates the Spinal Cord Injury Induced by Acute Trauma via Suppressing the Expression of Perforin" was retracted in 2022. Reason: concerns about the peer review.

Levetiracetam is an antiepileptic drug which can effectively improve the symptom of epilepsy via blocking the neurotransmitter release [10]. Recently, the therapeutic effect of levetiracetam on cerebral diseases induced by nerve injury has been proved by some researches. The reporter showed that levetiracetam can improve the cerebral neuronal injury induced by ischemic reperfusion via blocking the degranulation and perforin release of CD8+ T cells [11]. Our previous study showed that perforin which originated from CD8+ T cells can aggravate the injury of spinal cord injury via damaging the BSCB of the mouse models [12]. However, whether levetiracetam can improve the acute trauma of spinal cord remains vague.

This study attempted to verify the effect of levetiracetam on SCI and reveal whether levetiracetam could improve the symptom of SCI via inhibiting the expression of perforin.

## 2. Materials and Methods

### 2.1. Animal Models

C57BL/6J mice with age 7-8 weeks and the weight ranging from 17 to 22 g were selected as the subjects in this study; the SCI mouse models were established by Jackson Laboratory. The SCI mice were randomly divided into the control group and the levetiracetam group. After SCI intervention, the mice in the levetiracetam group were immediately fed with 180 mg/kg levetiracetam, while the mice in the control group were fed with 180 mg/kg saline. Moreover, all mice were cared and bred in the experimental animal center of Jinan University Medical College. The experiments were approved by the Commission for Animal Protection and Use of Jinan University.

### 2.2. SCI Model Establishment

The SCI mouse model establishment was performed with the spinal cord hitter manufactured by New York University. In brief, 1.25% tribromoethanol was injected into the T11 levels of the mice, and then, the related spinal dura mater of T11 levels was exposed. Subsequently, the T11 vertebral bodies of the mice were fixed and then struck with a 10 g impact rod dropped from 6.25 mm. After that, the models was tested via controlling bilateral hind limbs and the tail of the mice.

The article "Levetiracetam Attenuates the Spinal Cord Injury Induced by Acute Trauma via Suppressing the Expression of Perforin" was retracted in 2022. Reason: concerns about the peer review.

### 2.3. Basso Mouse Score

The hind motor functions of the mice were observed by Basso mouse score. In brief, the mice were placed on a flat surface for 5 min, and then, their hind limb abilities were observed. The scorning of the mice was performed following the principle of Basso mouse score ranging from 0 to 9, and the scores of the mice were positively related with abilities of the mice.

### 2.4. CatWalk-Assisted Gait Analysis

The walking coordination of the mice was assessed with the CatWalk XT gait analysis system. In short, the mice were placed in the dark, and their gait on a 50 cm glass flat path was recorded by CatWalk XT (Noldus). The regularity index was used to calculate the walking coordination of the mice. Moreover, the regularity index of the normal animals was 100%. The formula of regularity index is as follows: the number of normal step-sequence patterns multiplied by four and divided by total paw placement.

### 2.5. Macrophage Infiltration Analysis

1 mL of 3% fluid thioglycolate medium was used to treat the mice. After 3 days, the mice were intravenously injected with 2 × 10^6^ macrophages labeled by carboxyfluorescein diacetate-succinimidyl ester (CFSE). The sections of the tissues were stained with F4/80 antibody and then were observed under the fluorescence microscope.

### 2.6. Nissl Staining

For Nissl staining, the nerve cells of the mice were observed by Nissl staining. In brief, after dewaxing, the paraffin sections (5 *μ*m) of the spinal cord were stained with Nissl reagent at 56°C for 1 h. After that, the sections were washed with deionized water for 30 seconds. After polarization and dehydration, the sections were sealed with resinene and then used to observe the injury of nerve cells.

### 2.7. Cell Apoptosis Detection

The cell apoptosis was observed by TdT-mediated dUTP nick end labeling (TUNEL) staining. In brief, the cell was dripped and dried onto the slide and then treated with TdT enzyme reaction liquid at 25°C for 2-5 min. The slide was treated with washing and stopping reaction buffer at 37°C. After that, 0.05% DAB was added into the slide at 25°C for 3-6 min. The slide was then observed under a fluorescence microscope (magnification, ×100).

### 2.8. Western Blot

The abundance of perforin in the tissues was detected by western blot. In short, the total proteins in the tissues were extracted by RIPA lysis buffer (Beijing Nobleide Technology Co., Ltd., Beijing, China). The total proteins were quantified and then separated with SDS-polyacrylamide gel. After that, the proteins were transferred to polyvinylidene fluoride membranes by wet-transfer methods. Subsequently, the membranes were blocked with 5% fat-free milk for 2 hours and then were incubated with the primary antibodies including anti-perforin (ab256453, Abcam), Occludin (ab216327, Abcam), Claudin-5 (ab131259, Abcam), and anti-*β*-actin (ab179467, Abcam) at 4°C overnight. The membranes were washed with the TBST for three times and then were incubated with secondary antibodies for 2 hours. Finally, the proteins were quantified by a chemiluminescence detection system.

The article "Levetiracetam Attenuates the Spinal Cord Injury Induced by Acute Trauma via Suppressing the Expression of Perforin" was retracted in 2022. Reason: concerns about the peer review.

### 2.9. ELISA

The perforin and inflammatory factors including IL-4, G-CSF, GM-CSF, IL-1*β*, IL-6, MCP-1, IFN-*γ*, and TNF-*α* in the serum of SCI mice were measured with ELISA kits. The kits were purchased from Beijing Plilai Gene Technology Co., Ltd. (Beijing, China).

### 2.10. Statistical Analysis

All data in this study were analyzed and visualized with SPSS 21.0 and GraphPad Prism 8, respectively. The difference of the data was tested with a chi-squared test or ANOVA with Tukey's post hoc test. *P* < 0.05 represented that the difference was statistically significant.

## 3. Results

### 3.1. Levetiracetam Improved the Motor Functions of SCI Mice

To observe the effect of levetiracetam on the spinal cord injury of SCI mice models, levetiracetam was used to treat the SCI mice, and the BMS, CatWalk-assisted gait analysis, and motor-evoked potentials were used to observed the hind limb motor functions of the mice 6 weeks after SCI intervention. The results of BMS and CatWalk-assisted gait showed that compared with the SCI mice in the control group, the mice in the levetiracetam group exhibited better performances in Basso mouse score and walking coordination, which suggested that levetiracetam can effectively recover the nerve conduction of SCI mice (Figure 1, *P* < 0.01). Thus, those observations suggested that levetiracetam could effectively improve the dysfunction in the hind limb motor function of SCI mice.

### 3.2. Levetiracetam Alleviated the Spinal Cord Injury of SCI Mice

To directly observe the effect of levetiracetam on improving the injury of SCI mice, the study detected the conditions in horizontal sections of SCI mice in 6 weeks via Nissl staining. Nissl staining showed that more Nissl bodies were observed in the mice treated with levetiracetam compared with the mice in the control group 3 days after levetiracetam intervention (Figure 2(a), *P* < 0.01). Moreover, the TUNEL staining showed that levetiracetam remarkably reduced the apoptosis rate of the cells in the trauma area (Figure 2(b), *P* < 0.01). Those observations suggested that levetiracetam could effectively protect the spinal cord of mice from the injury.

The article "Levetiracetam Attenuates the Spinal Cord Injury Induced by Acute Trauma via Suppressing the Expression of Perforin" was retracted in 2022. Reason: concerns about the peer review.

### 3.3. Levetiracetam Relieved the BSCB Disruption of SCI Mice

The permeability of BSCB was observed by F4/80 staining, and levetiracetam can significantly reduce the numbers of macrophages transferred through the BSCB (Figure 3(a), *P* < 0.01). Besides, levetiracetam significantly restored the expression levels of Occludin and Claudin-5 in the vascular endothelial cells of the SCI mice 3 days after injury. Those observations suggested that levetiracetam can relieve the BSCB disruption of SCI mice (Figures 3(b) and 3(c), *P* < 0.01).

### 3.4. Levetiracetam Reduced the Inflammatory Reactions in SCI Mice

To investigate whether levetiracetam improved the spinal cord injury via regulating the inflammatory reactions of SCI mice, the expression level of the inflammatory factors was measured 3 days after levetiracetam intervention. The results showed that the levels of the inflammatory factors including IL-4, G-CSF, GM-CSF, IL-1*β*, IL-6, MCP-1, IFN-*γ*, and TNF-*α* significantly reduced in the SCI mice treated with levetiracetam (Figure 4, *P* < 0.01). Thus, it suggested that levetiracetam can prevent SCI of mice via inhibiting the inflammatory reactions.

### 3.5. Levetiracetam Prevented the Expression of Perforin in SCI Mice

To reveal the drug mechanism of levetiracetam, the expression level of perforin in injured tissues and serum of SCI mice was measured. In the results, the abundance of perforin was significantly downregulated in injured tissues of SCI mice treated with levetiracetam 3 days after levetiracetam intervention (Figure 5, *P* < 0.01). Thus, it suggests that levetiracetam inhibited the expression of perforin to block the progression of SCI.

## 4. Discussion

The injury of nerve cells can be a major reason for the formation and development of several central nervous system-related diseases, and the low regeneration ability of nerve cells may induce the irreversible motor dysfunction of the patients [13, 14]. BSCB plays a critical role in protecting the spinal cord away from macrophage-mediated inflammatory stress, and BSCB disruption can promote the deterioration of SCI. Levetiracetam has been proved to improve the ischemic reperfusion injury of cerebral nerve cells [15, 16]. However, few studies have revealed the function of levetiracetam in the acute trauma of the spinal cord. In this study, the therapeutic effect of levetiracetam on spinal cord injury was investigated via SCI mouse models.

The article "Levetiracetam Attenuates the Spinal Cord Injury Induced by Acute Trauma via Suppressing the Expression of Perforin" was retracted in 2022. Reason: concerns about the peer review.

The blocked nerve conduction is major reason leading to the impairment of motor functions of the patients with spinal cord injury. In this study, it was found that levetiracetam could effectively improve the hind limb motor functions, which involves the protection of nerve conduction and protection of the walking coordination of SCI mice. Macrophage-induced immune reaction plays a critical role in the progression SCI, and macrophage infiltration has been confirmed in the progression of SCI [17]. Strikingly, this study revealed that levetiracetam can effectively improve the inflammatory level in SCI mice, and the inflammatory factors such as IL-1*β*, GM-CSF, IFN-*γ*, and TNF-*α* were upregulated in SCI mice, unexceptionally. Levetiracetam has been found to significantly alleviate the inflammation in sciatic nerves and impede the electrophysiological alterations of diabetes mice [18]. Those proofs imply that levetiracetam may improve the SCI of the mice via inhibiting the inflammation reactions.

Macrophage infiltration can aggravate the injury of the spinal cord, which is related to BSCB dysfunction [19]. BSCB serves an important role in separating the nerve cells and macromolecular substances, which protects the stability of the central nervous system (CNS) [20]. Destruction of the BSCB or blood-brain barrier (BBB) has been proved to induce CNS injury or several neurodegenerative diseases [21]. Several studies have indicated that the destruction of BSCB can secondly induce the injury of the spinal cord and thus aggravate the symptom of SCI [22, 23]. In this study, levetiracetam distinctly restored the BSCB in vivo and decreased the permeability of BSCB of the mouse models induced by SCI. Claudin-5 and Occludin serve important roles in maintaining the permeability of BSCB, and the deficiency of Claudin-5 and Occludin has also been found in the brain injury induced by BSCB damage [24, 25]. Moreover, in a previous study, decreased Claudin-5 and Occludin have been also found in the SCI mice. In this study, levetiracetam significantly reversed the expression of the abundance of Claudin-5 and Occludin in BSCS of SCI mice. Thus, those proofs suggest that levetiracetam can improve the integrality of BSCS via supporting the expression of Claudin-5 and Occludin.

The study has revealed that CD8+ T cells could alter the permeability of BBB via releasing perforin and thus have a critical role in the formation of peptide-induced fatal syndrome [26]. In a previous study, it has been found that the CD8+ T cell knockout could remarkably improve the symptom of SCI mice, and the CD8+ T cells with perforin knockdown can also alleviate the spinal cord injury of the mice and restore the expression of Claudin-5 and Occludin [12]. In this study, it was found that levetiracetam extremely decreased the abundance of perforin in the CD8+ T cells and serum of SCI mice. Moreover, the study has indicated that levetiracetam can also relieve the acute cerebral injury induced by ischemic reperfusion via blocking the expression of perforin [11]. In this study, it was found that levetiracetam promoted the expression of Claudin-5 and Occludin in the BSCB of SCI mice. Thus, this study suggested that levetiracetam could improve the injury of blood-brain barrier by reversing the expression of Claudin-5 and Occludin.

The article "Levetiracetam Attenuates the Spinal Cord Injury Induced by Acute Trauma via Suppressing the Expression of Perforin" was retracted in 2022. Reason: concerns about the peer review.

In autoimmune enteric ganglionitis, the effect of CD8 T cells on neuronal destruction is perforin dependent [27]. Inflammatory stress has been confirmed as a major reason for myelin and neuronal injury. Moreover, the increased perforin may also mediate the poor prognosis of the patients with inflammatory cardiomyopathy [28]. Moreover, it was also found that levetiracetam could significantly inhibit the expression of perforin. Thus, those observations suggested that levetiracetam alleviates the inflammatory reactions to improve the progression of SCI via inhibiting CD8 T cell-derived perforin.

## Figures and Tables

**Figure 1:** Levetiracetam effectively improved the motor function of SCI mice. (a–c) CatWalk-assisted gait analysis for the mice 6 weeks after SCI intervention. (d) Basso mouse score for the mice 6 weeks after SCI intervention. ^∗∗^*P* < 0.01.

**Figure 2:** Levetiracetam effectively improved the acute trauma of SCI mice. (a) Nissl staining for the injury region of the mice 6 weeks after SCI intervention. (b) TUNEL staining for cell apoptosis in the injury region of the SCI mice 3 days after levetiracetam intervention. ^∗∗^*P* < 0.01.

**Figure 3:** Levetiracetam significantly alleviated the disruption of BSCB in SCI mice. (a) F4/80 staining of macrophages in the spinal cord of SCI mice 3 days after levetiracetam intervention. (b, c) The expression level of Occludin and Claudin-5 in the injury region of SCI mice at day 3 after injury. ^∗∗^*P* < 0.01.

**Figure 4:** Levetiracetam remarkably reduced the inflammatory reactions in SCI mice. (a) The heat map of inflammatory factors of mice after 24 hours of SCI. (b) The abundance of inflammatory factors in the serum of the mice after 24 hours of SCI. ^∗∗^*P* < 0.01.

**Figure 5:** Levetiracetam significantly suppresses the expression of perforin in the tissues and serum of SCI mice. (a, b) The abundance of perforin in the tissues of SCI mice. (c) The abundance of perforin in the serum of SCI mice 3 days after injury. ^∗∗^*P* < 0.01.

## Data Availability

Data to support the findings of this study is available on reasonable request from the corresponding author.
